The article "PRR15 Is a Novel Diagnostic and Prognostic Biomarker in Papillary Thyroid Cancer and Modulates the Tumor Microenvironment" was retracted in 2023. Reasons: suspected computer-generated content; unreliable results or conclusions; concerns about the data; concerns about the results or conclusions.

# PRR15 Is a Novel Diagnostic and Prognostic Biomarker in Papillary Thyroid Cancer and Modulates the Tumor Microenvironment

**DOI:** 10.1155/2022/3290479

**Published:** 2022-09-15

**Authors:** Lingli Wang, Xiaoqing Deng, Yi Chen, Yixia Zhao, Zhirong Li

**Affiliations:** ^1^Department of Breast and Thyroid Surgery, Daping Hospital, Army Medical University, Chongqing, China; ^2^Department of Nephrology, The First Affiliated Hospital of Chongqing Medical University, Chongqing, China; ^3^Department of Pharmacy, Chongqing University Cancer Hospital, Chongqing, China; ^4^Digestive Center, University-Town Hospital of Chongqing Medical University, Chongqing, China

## Abstract

Papillary thyroid cancer (PTC), accounting for more than 80 percent of all cases of thyroid cancer, is a form of a cancerous tumor that has a very favorable prognosis. However, patients diagnosed with PTC who are already in an advanced state have a dismal outlook. This study aimed to establish the diagnostic relevance of PRR15 expression in PTC patients as well as its levels in PTC samples and its connection with immune infiltrates. The TCGA and GEO datasets were combed through to obtain information on PTC patients. The “Limma” program was used to screen for differentially expressed mRNAs (DEMs), and the results were displayed using volcano plots and heat maps. The Wilcoxon test was used to examine the level of PRR15 expression in PTC patients in comparison with that of normal tissues. To study the connection between the immune infiltration level and PRR15 expression in PTC, the single-sample sequence set enrichment analysis (ssGSEA) from the R package was utilized. The expression of PRR15 was analyzed with RT-PCR in PTC cells and normal cells. In order to evaluate the diagnostic significance of PRR15 expression, ROC assays were carried out. Experiments using CCK-8 were carried out to investigate the impact that PRR15 knockdown could have on the proliferation of PTC cells. In this study, 17 overlapped DEMs between PTC specimens and normal specimens were identified, including MPPED2, IPCEF1, SLC4A4, PKHD1L1, DIO1, CRABP1, TPO, TFF3, SPX, TCEAL2, ZCCHC12, SYTL5, PRR15, CHI3L1, SERPINA1, GABRB2, and CITED1. Our attention focused on PRR15 which was highly expressed in PTC specimens as compared with nontumor specimens. PRR15 had an AUC value of 0.926 (95% CI 0.902–0.950) for PTC based on TCGA datasets. Pan-cancer assays suggested PRR15 as an oncogenic gene in many types of tumors. Moreover, we found that PRR15 expression was positively correlated with eosinophils, NK cells, NK CD56bright cells, IDC, macrophages, DC, mast cells, and Th1 cells. Further investigations with CCK-8 demonstrated that inhibiting PRR15 resulted in a decrease in the proliferation of PTC cells. Overall, PRR15 was confirmed to be a biomarker for PTC patients and a predictor of response to immunotherapy.

## 1. Introduction

Thyroid cancer, which is the most prevalent kind of endocrine malignant tumor, is increasing at a rate of one percent per year around the world and has shown a rapid increase in morbidity [1]. Papillary thyroid carcinoma (PTC) is the most common kind of thyroid cancer [2]. It accounts for around 60–70 percent of all thyroid cancers, and it most frequently affects women in their fourth and fifth decades of life [3]. Many PTCs are well differentiated and have a low risk of recurrence, but a small proportion of tumors reveal heterogeneity with more aggressive variations [4, 5]. Because so little is known about the potential mechanisms of aggressive variations, the therapy for PTC cases is frequently insufficient or less than ideal. Therefore, diagnostic and prognostic biomarkers are desperately needed as soon as possible because these would assist doctors in implementing early and suitable steps for maximum treatment benefit.

PTCs encompass several subtypes, including a classical variant of tall cell variant of PTC (tPTC), follicular variant of PTC (fVPTC), and papillary thyroid carcinoma (cPTC) [6]. According to the established criteria recognized by the World Health Organization, other histologic variations include diffuse sclerosing, columnar, and others [7]. It is possible that the prognosis for various histologic subtypes of PTC will be varied. Based on the developing idea of “precision medicine,” recent years have seen significant advancements in molecular pathology detection tools and tailored therapy, both of which have contributed to a dramatically increased overall survival rate for patients diagnosed with PTC [8, 9]. In the field of precision medicine, the genes that are most responsible for the development of cancer could be applied as therapeutic targets [10]. Several molecules are involved in adenocarcinoma including the anaplastic lymphoma kinase gene, echinoderm microtubule-associatedprotein-like gene, and epidermal growth factor receptor mutations [11, 12]. Even while molecularly targeted medicines have shown promising outcomes in clinical testing, there is still a long way to go before patients diagnosed with PTC may be cured, particularly due to the evolution of drug resistance. Therefore, patients diagnosed with PTC require the identification of more accurate indicators for diagnosis and prognosis of PTC patients.

Immunotherapy has recently garnered a great deal of attention as a potentially effective treatment for a variety of malignancies [13]. Immune checkpoint inhibitors (ICIs) are another name for T cell-based immunotherapy [14]. Immunotherapy and associated treatments targeting T cell exhaustion indicators can improve the long-term survival of tumor patients by increasing antitumor immunity, which has exhibited considerable therapeutic benefit in immunogenic cancers such as liver cancer, glioma, rectal cancer, renal cell carcinoma, and melanoma [15, 16]. However, the therapy provided by ICIs is not effective for all patients. The varying response is also connected with the genetic characteristics of the patients, such as the tumor microenvironment (TME) [17]. Research conducted throughout time has accumulated evidence that tumor cells can alter the TME to function as contributors that assure fast cell proliferation [18]. The dynamic alteration of molecular and cellular processes in TME relays on the interactions between tumor cells and immune cells, which highlights the role of TILs in the context of protumorigenic inflammation and anticancer immunosurveillance.

In this study, we analyzed GEO datasets and identified several differentially expressed mRNAs (DEMs) in PTC. Among them, our attention focused on proline-rich 15 (PRR15). PRR15 is a nuclear protein with a low-molecular weight that is expressed by the trophoblast in the early stages of pregnancy. The death of the embryo on day 15 of gestation was caused by lentivirus-mediated reduction of PRR15 mRNA in ovine trophectoderm [19]. This provides solid evidence that PRR15 expression is crucial during this precarious window of development. In recent years, PRR15 has been reported to be dysregulated in several tumors, such as breast cancer, esophageal cancer, and human gastrointestinal tumors [20, 21, 22]. However, its specific function and clinical significance were rarely reported. In this study, we aimed to explore the prognostic value of PRR15 expression and its association with the tumor microenvironment.

## 2. Methods

### 2.1. Cell Culture and Cell Transfection

The human normal thyroid epithelial cell line (Nthy-ori 3-1) and the PTC cell lines (FTC-133, 8505C, TPC1, and BCPAP) were purchased. All of the cell lines were kept alive in DMEM (Invitrogen, China), which was supplemented with 10 percent FBS (PAN, China). The cells were cultured at a temperature of 37°C in an atmosphere that contained 5 percent carbon dioxide.

RiboBio (Guangzhou, China) was the supplier for both PRR15 small interfering RNA (siRNA) and negative control siRNA (si-NC). The Lipofectamine 2000 reagent (manufactured by Invitrogen) was used to achieve cell transfection in accordance with the manufacturer's instructions.

### 2.2. qRT-PCR Analysis

In order to get total RNA from TPC tissues or cells, the TRIzol (Invitrogen, USA) kit was used, and the process followed the procedure provided by the manufacturer. To perform reverse transcription on the shared gene and miRNA, the HiScript® III 1st Strand cDNA Synthesis Kit (+gDNA wiper) (Vazyme, China) was used. To carry out reverse transcription of miRNA, a First Strand cDNA Synthesis Kit (by stem-loop) (Vazyme, China) was utilized. Amplification of the target genes was done by qPCR, and the ChamQ-Universal-SYBR qPCR Master Mix was applied for the quantification (Vazyme). The following describes the cycle conditions for RT-qPCR: first, denaturation was performed at 95°C for ten minutes, followed by forty cycles of denaturation at 95°C for fifteen seconds and annealing/elongation at 60°C for sixty seconds each. Internal controls were determined using either GAPDH or U6. The 2-CT technique was utilized in order to carry out the task of determining the extent to which the target gene was amplified. The involved primers were as follows: PRR15 forward: 5′-GCTCACCAACAGCAGAAAGAA-3′, PRR15 reverse: CGGATTTGTCCCCGTATAACTTG; GAPDH forward: 5′- ACAACTTTGGTATCGTGGAAGG-3′, GAPDH reverse: 5′-GCCATCACGCCACAGTTTC-3′.

### 2.3. Cell Counting Kit-8 (CCK-8) Experiment

We used a commercial product called CCK-8 to determine the vitality of the cells. PTC cells with a density of 5 × 10^3^ cells per well were seeded onto 96-pore dishes, and a further 10 *µ*l of CCK-8 solution was added for an additional two hours of growth. It was determined that each well had an absorbance of 450 nm.

### 2.4. Data Processing

The datasets for papillary thyroid carcinoma, also known as THCA, were gathered from two different platforms. There was a search conducted in The Cancer Genome Atlas (TCGA) database (https://portal.gdc.cancer.gov/repository) using the THCA database level 3 count. The values in the datasets that are part of TCGA have been converted into transcripts per million (TPM). The THCA clinical data were gathered by utilizing the UCSC Xena browser, which may be found online at https://xenabrowser.net/. In this retrospective study, we only considered patients who had primary tumors and who had not previously been treated with neoadjuvant chemotherapy or radiation. Their survival data, together with their clinicopathological, genetic, and epigenetic information, were downloaded for a secondary study. The datasets containing 510 tumor samples and 58 normal samples were utilized in this research project. The clinical information of all PTC is shown in Table 1. Two different Gene Expression Omnibus (GEO) datasets were examined for this study. Downloads were made up of the series matrix files of GSE33630 (which had 60 cases of thyroid cancer and 45 cases of normal tissue) and GSE3678 (which contained 7 cases of papillary thyroid carcinoma and 7 cases of normal tissue). Afterwards, the gene expression in PTC and normal thyroid tissue was compared using the normalized values of the genes.

### 2.5. Identification of Differentially Expressed mRNA (DEMs) in PTC

The raw count data were first transformed into log2 form after being standardized with the transcripts per million (TPM) method. The next step was the annotation of 19654 protein-coding genes. “Limma,” in its version 3.36.2 for the R programming language, was used in the DEM calculations [23]. DEMs that had an absolute log2 fold change (FC) of >1 and an adjusted *P* value of <0.05 were taken into consideration for further study.

### 2.6. Estimation of TME Immune Infiltration

Bindea et al. provided us with the gene set that could be used to represent many sorts of immune cells that infiltrated the tissue. After that, ssGSEA was applied to compute the number of immune cells present based on the expression of the reference gene contained within the gene set that was obtained from the transcriptomic data. 24 types of immune cells were enrolled in our study.

### 2.7. Statistical Analyses

R software version 3.5.3 was used to carry out the statistical analyses. Student's *t*-test and the chi-square test were used to do a comparison between the two groups. The ROC was an invaluable tool in establishing the diagnostic value of PRR15 for PTC patients. Kaplan–Meier analysis and the log-rank test were performed to identify survival differences in TPC patients. A heat map and volcano map were used to show the DEMs between PTC specimens and nontumor specimens. A *p* < 0.05 was considered to indicate a statistically significant difference.

## 3. Results

### 3.1. Identification of DEMs between PTC Samples and Normal Samples

In the first step of our research, we examined the GSE3678 datasets, which contained both PTC and normal samples. The limma program was utilized in order to perform an analysis on the DEMs of the metadata. 574 DEMs were collected: 244 genes were upregulated and 330 genes were downregulated (Figure 1(a)). Similarly, we analyzed GSE33630 datasets which included 60 tumor samples and 45 normal samples, and 1229 mRNAs were collected in which 615 mRNAs were upregulated and 614 mRNAs were downregulated (Figure 1(b)). To further screen the critical functional genes involved in PTC progression, we used a heat map to show the top 20 dysregulated mRNAs between PTC samples and normal samples in GSE3678 (Figure 1(c)) and GSE33630 (Figure 1(d)). Finally, 17 overlapped DEMs were identified, including MPPED2, IPCEF1, SLC4A4, PKHD1L1, DIO1, CRABP1, TPO, TFF3, SPX, TCEAL2, ZCCHC12, SYTL5, PRR15, CHI3L1, SERPINA1, GABRB2, and CITED1 (Figure 1(e)).

### 3.2. The Distinct Upregulation of PRR15 in PTC and Its Diagnostic Value

Among the 17 genes, our attention was focused on PRR15 which was highly expressed in PTC specimens compared with nontumor specimens in both GSE3678 (Figure 2(a)) and GSE33630 datasets (Figure 2(b)). Then, we analyzed TCGA datasets and also confirmed PRR15 as an overexpressed gene in PTC (Figures 2(c) and 2(d)). In addition, the results based on TCGA datasets and GTEx data were in line (Figure 2(e)). Then, we further explored the possible diagnostic potential of higher PRR15 expression in screening PTC patients. As presented in Figure 2(f), PRR15 had an AUC value of 0.926 (95% CI 0.902–0.950) for PTC based on TCGA datasets. Moreover, a similar finding was observed based on TCGA datasets and GTEx data (Figure 2(g)).

### 3.3. The mRNA Expression of PRR15 in Cancers

Data from the TCGA datasets showed that PRR15 expressions were distinctly higher in BRCA, CHOL, LIHC, LUSC, PAAD, STAD, THCA, and UCEC, while its expression was distinctly lower in COAD, KICH, KIRC, KIRP, and PRAD (Figure 3(a)). Based on TCGA and GTEx databases, we found that more tumor specimens exhibited a higher level of PRR15 (Figure 3(b)). Thus, our findings suggested that PRR15 may exhibit a different role based on the types of tumors. According to our results, its main function may be a tumor promotor.

### 3.4. Association between PRR15 Levels and Clinicopathological Parameters of PTC

We studied the relationship between PRR15 levels and the clinicopathological features of PTC so that we might gain a better understanding of the clinical relevance of PRR15 expression in patients with PTC. We did not find distinct differences between the PRR15 expression and several clinicopathological parameters of PTC, including age (Figure 4(a)), gender (Figure 4(b)), T stage (Figure 4(c)), and M stage (Figure 4(d)). However, we found that PTC specimens with advanced N stage exhibited a higher level of PRR15 than those with low N stage (Figure 4(e)).

### 3.5. PRR15 Expression Is Correlated with Immune Infiltration Level in PTC

As shown in Figure 5(a), we found that PRR15 expression was positively correlated with eosinophils, NK cells, NK CD56bright cells, IDC, macrophages, DC, mast cells, and Th1 cells. The representative diagram of the correlation analysis between PRR15 expression and immune-infiltrating cells is shown in Figure 5(b).

### 3.6. Knockdown of PRR15 Suppressed the Proliferation of PTC Cells

We used RT-PCR to see if PRR15 expression was abnormal in PTC cells, Nthy-ori 3-1 cells had decreased PRR15 expression compared to PTC cell lines FTC-133, 8505C, TPC1, and BCPAP cells (Figure 6(a)). Loss-of-function experiments in vitro were carried out to examine the biological significance of PRR15 in PTC cells. An oligonucleotide (si-PRR15) transfection reduced the expression level of PRR15 considerably in 8505C and TPC1 cells (Figure 6(b)). CCK-8 assays showed that PRR15 knockdown significantly reduced 8505C and TPC1 cell growth when compared to negative control transfection (Figures 6(c) and 6(d)).

## 4. Discussion

PTC has been shown to correlate with external radiation exposure, dietary iodine content, and the subsequent disturbance of thyroid stimulating hormone (TSH) levels throughout the course of the past few decades [24, 25]. Today, a rising number of investigations are beginning to focus on acquired genetic alterations that can discriminate paratumor normal tissue from PTC specimens. The early diagnosis of PTC patients is very important, which can help doctors develop the best treatment plan. As a result, our understanding of the molecular etiology of PTC has significantly expanded. In clinical settings, a number of other biomarkers, such as RET/PTC rearrangement, PAX8-PPAR rearrangement, BRAF mutations, and RAS mutations, have been employed [26, 27]. Therefore, screening sensitive biomarkers would be of tremendous value for the customized prevention and treatment of patients suffering from PTC.

First, we analyzed the GSE3678 and GSE33630 datasets. DEMs were analyzed by the use of the limma package. We overlapped 17 DEMs, including MPPED2, IPCEF1, SLC4A4, PKHD1L1, DIO1, CRABP1, TPO, TFF3, SPX, TCEAL2, ZCCHC12, SYTL5, PRR15, CHI3L1, SERPINA1, GABRB2, and CITED1. Among the above DEMs, several of them have been reported to be involved in the progression of several tumors. For instance, Zhang et al. reported that in PTC, miR-222-3p had a high level of expression, while SLC4A4 had a low level of expression. PTC cells were shown to benefit from the presence of miR-222-3p in terms of their ability to proliferate, invade, and migrate. These stimulatory effects of miR-222-3p were able to be inhibited by SLC4A4, as expected [28]. Lin et al. showed that TFF3 expression was shown to be increased in PTC tissue, and this increase in expression was associated with lymph node metastasis, pathological grade, and snail expression. TPC1 cells were significantly hindered in their capacity for proliferation, adhesion, colony formation, migration, and invasion after having their TFF3 levels significantly reduced. The findings showed that TFF3 might potentially activate the MAPK/ERK signaling pathways mechanically [29]. Wang and his group reported that the ZCCHC12 gene was shown to be significantly amplified in primary PTC cancers. Overexpression of ZCCHC12 was found to correlate with lymph node metastases in both cohorts. In trials conducted in vitro, a decrease in ZCCHC12 expression led to a considerable inhibition of PTC cell colony formation, motility, and invasion [30]. These findings suggested DEMs as important regulators in progression of PTC. However, the expression and function of PRR15 have not been investigated in PTC. In this study, we first reported that PRR15 expression was distinctly increased in PTC cell lines. PRR15 had an AUC value of 0.926 (95% CI 0.902–0.950) for PTC based on TCGA datasets. Moreover, a similar finding was observed based on TCGA datasets and GTEx data, which confirmed the diagnostic value of PRR15 in screening PTC specimens from normal specimens. In addition to this, we were able to demonstrate that inhibiting PRR15 in PTC cells led to a reduction in their rate of proliferation. In general, our research indicated that PRR15 may serve as both a new diagnostic biomarker and an oncogene in individuals with PTC.

Equally as crucial, our research revealed the connection between PRR15 expressions and immune infiltration in PTC by utilizing ssGSEA and Spearman correlation. We found that PRR15 expression was positively correlated with eosinophils, NK cells, NK CD56bright cells, IDC, macrophages, DC, mast cells, and Th1 cells. Many tumors, including bladder cancer, lung cancer, and melanoma, have Th1/Th2 balanced drift in the body, and Th2 cells are often dominant, which may be related to the immune escape of tumors [31, 32]. There is a growing trend in research to try and develop medications and technologies that can either stabilize the Th1/Th2 balance or bring about a reversal of it [33]. For example, the use of cytokines or cytokine antagonists in the therapy of cancers and other disorders to reestablish a healthy balance between Th1 and Th2 cells: cytokines produced by Th1 cells have the ability to shift the Th1/Th2 equilibrium toward a Th1 state while simultaneously decreasing the dominant expression of Th2 cells. The opposite impact was produced by Th2 cytokines. Patients who have a higher than average number of infiltrating DC in many different kinds of cancers have a better prognosis than patients who do not have a higher than average number of these cells [34]. There is a close association between DC and the occurrence and progression of cancers [35, 36]. The generation of a cellular immune response that is dominated by CD8+ T cells is essential to the production of an effective antitumor immune response. These cells are also the foundation of DC as an immunotherapy.

There are still some limitations in the current study. First, this investigation looked back at previous events. Therefore, in the future, there ought to be a prospective study carried out in order to eliminate the analysis bias that is linked with studies that are retrospective. Second, since the number of healthy subjects who participated in the study to serve as controls was significantly lower than the number of patients who participated in the study to have cancer, additional research was required to ensure that there was an equal distribution of patients and healthy subjects among the samples. Last, the purpose of this work, which was carried out in vitro, was to investigate the possible role that PRR15 expression plays in PTC progression. To validate our findings, we needed to conduct additional tests on living animals.

## 5. Conclusion

In our study, PRR15 was shown to be an important molecular biomarker with diagnostic significance and may have a major impact on the modulation of immune infiltration in PTC. This research work provides promising visions for future research to elucidate the molecular pathogenesis of PTC as well as its clinicopathological importance. It is necessary to conduct randomized clinical trials in addition to more research studies to investigate the underlying mechanism and clinical applications for PTC patients.

## Figures and Tables

**Figure 1:** Identification of the DEMs between PTC specimens and nontumor specimens. (a)-(b) The number of DEMs found in the GSE3678 and GSE33630 datasets is displayed using volcano charts. (c)-(d) The top 20 DEMs found in the GSE3678 and GSE33630 datasets are displayed on a heat map. (e) The genes that are shared by both GSE3678 and GSE33630 datasets are depicted in a Venn diagram.

**Figure 2:** The expression of PRR15 in PTC patients and its diagnostic value. ((a)-(d)) PRR15 expression distinctly increased in PTC specimens compared with nontumor specimens in (a) GSE3678, (b) GSE33630, and (c)-(d) TCGA datasets. (e) The upregulation of PRR15 in PTC patients further confirmed in TCGA and GTEx data. (f)-(g) ROC assays applied to determine the diagnostic value of PRR15 expression in screening PTC specimens from nontumor specimens in TCGA or TCGA and GTEx data.

**Figure 3:** Expression level of PRR15 in different cancer types from (a) TCGA or (b) TCGA and GTEx data.

**Figure 4:** The association between PRR15 expression and clinicopathological parameters of PTC, including (a) age, (b) gender, (c) T stage, (d) M stage, and (e) N stage.

**Figure 5:** The expression level of PRR15 is related to the immune infiltration in the tumor microenvironment. (a) The amount of PRR15 expression shown to have a correlation with the relative abundances of 24 immune cells. The magnitude of the dots is representative of the absolute value of Spearman (R). (b) A diagrammatic representation of the correlation analysis performed between PRR15 expression and immune-infiltrating cells.

**Figure 6:** PRR15 overexpressed in PTC and its knockdown suppressed the proliferation of PTC cells. (a) In order to establish the level of PRR15 expression in FTC-133, 8505C, TPC1, and BCPAP cells, RT-PCR analysis is utilized. (b) The expression of PRR15 distinctly decreased in TPC1 and 8505C cells after the transfection of si-PRR15. (c)-(d) CCK-8 experiments applied to examine the function of PRR15 knockdown on TPC1 and 8505C cells. The experiments are repeated three times and each experiment is triplicated.

**Table 1:** Association of PRR15 with clinicopathological characteristics of PTC patients.

Characteristics	The low expression of PRR15	The high expression of PRR15	*P*
*N*	255	255	
Gender, *n* (%)			0.691
Female	183 (35.9%)	188 (36.9%)	
Male	72 (14.1%)	67 (13.1%)	
Age, *n* (%)			0.723
≤45	118 (23.1%)	123 (24.1%)	
>45	137 (26.9%)	132 (25.9%)	
M stage, *n* (%)			0.505
M0	138 (46.8%)	148 (50.2%)	
M1	3 (1%)	6 (2%)	
N stage, *n* (%)			0.025
N0	123 (26.7%)	106 (23%)	
N1	99 (21.5%)	132 (28.7%)	
T stage, *n* (%)			0.500
T1	65 (12.8%)	78 (15.4%)	
T2	85 (16.7%)	82 (16.1%)	
T3	89 (17.5%)	86 (16.9%)	
T4	14 (2.8%)	9 (1.8%)	
Age, median (IQR)	48 (35.5, 60)	46 (34, 56)	0.096

## Data Availability

The databases generated during the current study are available from the corresponding author upon request.
